# Linc00261 Inhibited High-Grade Serous Ovarian Cancer Progression through miR-552-ATG10-EMT Axis

**DOI:** 10.1155/2022/9450353

**Published:** 2022-04-12

**Authors:** Lin Wang, Hongcai Wang, Jiuwei Chen

**Affiliations:** Gynecology Department, Zibo Maternal and Child Health Hospital, NO.66 North Tianjin Road, Zibo, Shandong Province 255000, China

## Abstract

In recent years, long non-coding RNAs (lncRNAs) play an important role in a multitude of pathways across species; however, their functions are still unknown. In this study, we demonstrate that Linc00261 is downregulation in high-grade serous ovarian cancer (HGSOC) and can inhibit cell proliferation and migration of high-grade serous ovarian cancer cells. We further validate the targeting interactions among Linc00261, miR-552, and ATG10. Interestingly, they all play important roles for regulating epithelial-mesenchymal transition (EMT) progression. Collectively, these findings suggest that Linc00261, a mediator of EMT progression, can target oncogenic miR-552, elevating ATG10 expression, to prevent high-grade serous ovarian cancer tumorigenesis and may serve as a potential novel therapeutic target.

## 1. Introduction

Ovarian cancer (OC) is a kind of malignant tumor of ovarian tumor, which refers to the malignant tumor growing on the ovary. Among them, 90%~95% are primary ovarian cancer, and the other 5%~10% are primary cancers in other parts that metastasize to the ovary. Due to the lack of symptoms in the early stage of ovarian cancer, even if there are symptoms, it is not specific, and the role of screening is limited, so the early diagnosis is more difficult. 60%~70% of patients are in the advanced stage at the time of treatment, and the curative effect of advanced cases is poor. Therefore, although the incidence rate of ovarian cancer is lower than that of cervical cancer and endometrial cancer, the third place is gynecologic malignancies, but the mortality rate is higher than that of cervical cancer and endometrial cancer. The main causes include continuous ovulation, environmental and other factors, and genetic factors [1].

High-grade serous ovarian cancer (HGSOC) is believed to come mainly from secretory cells in the fallopian tube, from where there is no obstacle to peritoneal spread [2]. HGSOC has the tropism of omental fat and can be used as an energy source. The inability to detect the disease in early diagnosis is one of the main factors for the higher mortality of HGSOC patients [3]. Studies have shown that only about 13% of serous ovarian cancer cases are diagnosed in stage I or II [4]. In fact, the vast majority of cases are usually diagnosed in the distant metastasis stage, which greatly affects the individual's prognosis [5–9]. So it is necessary and urgent to explore the mechanism of the onset, development, and metastasis of HGSOC.

Non-coding RNAs account for about 98% of all transcripts in the human genome, and most of non-coding RNAs are long non-coding RNAs [10], which commonly exhibit tissue-specific expression patterns and are associated with multiple functions [11–14]. Recently, increasing evidences indicate that many lncRNAs are deregulated in cancer and implicated in almost all hallmarks of cancer [15–28]. As to HGSOC, many lncRNAs are dysregulated. NEAT1 contributes to HGSOC tumorigenesis via targeting miR-506 [29]. LncRNA MEG3 (MEG3 is an imprinted gene located at 14q32 that encodes a lncRNA, and the decreased MEG3 expression has been reported in multiple cancer tissues) is decreased in HGSOC and is a hallmark for tumor progression in HGSOC [30]. A newly discovered lncRNA, LINC00261, has been found to act as a suppressive regulator in several cancers including colon cancer [31], non-small cell lung cancer [32], gastric cancer [33], and hepatocellular carcinoma [34] via various molecular mechanisms. However, it remains unclear whether Linc00261 (long intergenic non-protein coding RNA 261, a recently discovered lncRNA, is abnormally expressed in a variety of human malignancies) plays an indispensable function in the development of HGSOC disease. In this study, we discovered the expression level of Linc00261 was lower in HGSOC tissues than normal tissues. In addition, Linc00261 knockdown elevated HGSOC cell proliferation and migration capacity. Functional experiments revealed Linc00261 directly bound to inhibit miR-552 (miR-552 is a small non-coding RNA located on chromosome 1p34.3, and its expression level is significantly upregulated in tissues or cells of various tumors) expression and increase ATG10 expression, eventually suppressing HGSOC tumorigenesis.

## 2. Patients and Methods

### 2.1. Clinical Samples

A total of 23 pairs of frozen HGSOC tissues and normal tissues were randomly obtained with informed consent from patients in Zibo Maternal and Child Health Hospital. Ethical consent was granted from Zibo Maternal and Child Health Hospital. Tissues were stored in liquid nitrogen for use. The age of the control group was 39-66 years old, with an average age of (45.26 ± 1.36) years. The educational level: 8 patients with college degree or above and 22 patients with college degree or below; age of observation group from 40 to 69 years old, the average age was (45.34 ± 1.43) years old. Educational level: 9 patients with college degree or above and 21 patients with college degree or below. There was no statistical significance between the two groups in terms of basic data (age, education level) (*P* > 0.05).

### 2.2. Cell Cultures and Treatment

OVCAR3, OVCAR4, SNU119, CAOV4, CAOV3, and FTSEC were cultured in 1640 or DMEM medium (Invitrogen) supplemented with 10% fetal bovine serum at 37°C in an atmosphere containing 5% CO2.

### 2.3. Plasmid Construction, Small Interfering RNA (siRNA) Synthesis, and Transfection

The full-length and mutation-length of LINC00261 were PCR-amplified by Thermo Scientific Phusion Flash High-Fidelity PCR Master Mix (Thermo) and subcloned into the EcoRI and XhoI sites of the pcDNA3.1 vector (Invitrogen), named pcDNA3.1-LINC00261-wt and pcDNA3.1-linc00261-mut, respectively.

Plasmids, siRNAs, and miRNAs were transfected into cancer cells using Lipofectamine 2000, RNAiMAX (Invitrogen) according to the manufacturer's protocol.

miR-552 inhibitors (5′ − CCAACAGGCAAAAGGUUAAAC − 3′),

miR-552 mimics (5′ − GUUUAACCUUUUGCCUGUUGG − 3′), and negative controls (5′ − UCACAACCUCCUAGAAAGAGUAGA − 3′)

siLINC00261-1 (5′ − CCAAUAGACCAACAGCCAU − 3′),

siLINC00261-2 (5′ − GAAAGCUGUAGCCAUUCAA − 3′), and

siNC (ACGUGACACGUUCGGAGAA)

### 2.4. RNA Extraction and Real-Time qPCR Analysis

Total RNA was isolated from cancer cell lines using Trizol reagent (Invitrogen) in accordance with the manufacturer's instructions. RNA was reversely transcribed into first-strand cDNAs by using the TIANScript RT kit (Tiangen Biotech Co., Ltd., Beijing, China). Real-time qPCR was performed using TaqMan Human microRNA assay (Applied Biosystems) for miRNA analysis and SYBR Green (Takara) for mRNA analysis.

The primer sequences were as follows:

Linc00261 forward primer: 5′ − TCAGATTGCTCCTGGACACTT − 3′,

reverse primer: 5′ − GGACCATTGCCTCTTGATTAG − 3′;

Snail forward primer: 5′ − CTTCGCTGACCGCTCCAACC − 3′,

reverse primer: 5′ − GGAGCAGGGACATTCGGGAGA − 3′;

Slug forward primer: 5′ − GGCTCATCTGCAGACCCATT − 3′,

reverse primer: 5′ − TGCTACACAGCAGCCAGATT − 3′;

N-cadherin forward primer: 5′ − AAGGCGTTATGTGTGTATCTTC − 3′,

reverse primer: 5′ − TGGAAAGCTTCTCACGGCAT − 3′;

E-cadherin forward primer: 5′ − TTCAAAGTGGGCACAGATGGT − 3′,

reverse primer: 5′ − TAGGTGGAGTCCCAGGCGTA − 3′;

miR-552 forward primer: 5′ − GTTTAACCTTTTGCCTGTTGG − 3′,

reverse primer: 5′ − CGAACGCTTCACGAATTTG − 3′,

ATG10 forward primer: 5′ − TACGCAACAGGAACATCCA − 3′,

reverse primer: 5′ − AACAACTGGCCCTACAATGC − 3′,

ꞵ-actin gene as internal reference, forward primer: 5′ − AGGCCAA CCGCGAGAAGATG − 3′, reverse primer: 3′ − CACACGGAGTACTTG CGCTCAG − 5′.

### 2.5. Cell Proliferation

Cell viability was measured by Cell Counting Kit-8 method (Dojindo Laboratories). For cell proliferation assays, a total of 2,000 cells were seeded into 96-well plates. After 24 hours, cell proliferation was assessed according to the manufacturer's protocol. The cell proliferation curves were plotted using the absorbance at each time point. The experiment was repeated for 3 times.

### 2.6. Transwell Cell Migration Assay

The 8 *μ*m pore size membrane was used to perform the experiments (Millipore, Bedford, USA). After transfection, cells were suspended in serum-free medium, then seeded into the upper chamber with 2 × 10^4^ cells and cultured at 37°C for 1 day. The lower compartments were filled with medium containing 10% FBS. After 24 h of incubation, the cells migrated to the bottom surface of the membrane were stained with 0.5% crystal violet, examined by microscopy. We randomly selected 6 fields in each sample to calculate the number of cells passing through the membrane (100x). The experiment was repeated 3 times.

### 2.7. Western Blot Analysis

The cell samples were lysed in RIPA buffer, boiled with 1∗SDS loading buffer, then samples were separated on 10% SDS-PAGE and transferred to polyvinylidene fluoride (PVDF) membranes (Millipore, USA). The membranes were incubated with specific antibodies against Slug, Twist1, E-cadherin, and N-cadherin overnight at 4°C. GAPDH was used as an internal control. All antibodies were purchased from Abcam (USA).

### 2.8. Luciferase Reporter Assay

Luciferase activities were tested using a PmirGLO Dual-Luciferase Expression Vector (Promega, Madison) according to the manufacturer's instructions. LINC00261-WT or LINC00261-MUT was cotransfected with miR-552 mimics into cancer cells using Lipofectamine 2000 when the cells reached 60% confluence. Luciferase activity in each group was tested and normalized to Renilla.

### 2.9. Animal Experiment

Twelve male BALB/C nude mice (5 weeks of age) were randomly divided into two groups. 5∗10^^6^ OVCAR3 stable cells were subcutaneously injected into the flank of mice in 100μl HBSS. Tumor size was measured once per week and the tumor volume was calculated as 1/2 *LW*^2^, where *L* and *W* are the largest and the smallest perpendicular tumor diameter, respectively.

### 2.10. Statistical Analysis

GraphPad Prism software was used to conduct the statistical analysis (La Jolla, CA, USA). The data were expressed as mean ± SD by 3 independent assays. t-test was used for measuring comparisons between these groups. *P* < 0.05 was considered statistically significant. When representative figures are shown, these are representative of three independent repeats.

## 3. Result

### 3.1. Linc00261 Was Down-Expressed in HGSOC

To explore the clinical role of Linc00261 in HGSOC, the expression levels of Linc00261 were determined by taking advantage of 23 pairs of HGSOC's tissue via qRT-PCR assay. Linc00261 was significantly downregulated in HGSOC tissue compared to adjacent non-tumor tissues (Figure 1(a)). It was also detected that Linc00261 has obviously lower expression in HGSOC cell lines (OVCAR3, OVCAR4, SNU119, CAOV4, and CAOV3) compared with normal ovarian epithelial cell line (FTSEC) [35] (Figure 1(b)). To further validate the relationship between Linc00261 and clinicopathologic factors, the data showed that low level of Linc00261 expression was also associated with lymph node metastasis (Figure 1(c)).

### 3.2. Linc00261 Suppressed the Proliferation and Migration of HGSOC Cells

We further evaluated the correlation between Linc00261 and HGSOC's malignant phenotype. CAOV3 and OVCAR3 are p53-mutant cell lines, therefore molecularly considered to be HGSOC [35, 36]. So CAOV3 was selected to silence Linc00261 and OVCAR3 was chosen to transfect with pcDNA-Linc00261. CCK-8 test showed that Linc00261 knockdown elevated the proliferative ability of HGSOC cells (Figure 2(a)). The migration capacity by transwell assay revealed that knockdown of Linc00261 accelerated the migration of HGSOC cells (Figure 2(b)). Conversely, overexpression of Linc00261 inhibited HGSOC cell proliferation and migration (Figures 2(c) and 2(d)). Furthermore, OVCAR3 cells stably overexpressing Linc00261 were used to examine the function on tumorigenesis in vivo. The results showed that Linc00261 group restrained tumor weights and volumes markedly compared with control group (Figures 2(e)–2(g)). Therefore, our data suggested that Linc00261 inhibited HGSOC progression.

### 3.3. Linc00261 Regulated Epithelial-Mesenchymal Transition (EMT) Progression of HGSOC

It has been reported that Linc00261 suppresses epithelial-mesenchymal transition (EMT) progression in several cancers, such as gastric cancer and non-small cell lung cancer. So we want to know whether Linc00261 affects EMT progression in HGSOC cells. There was a noticeable change in mRNA expression of EMT hallmarks via knockdown of Linc00261. Slug, Twist1, and N-cadherin expression was upregulation; E-cadherin expression was downregulation (Figure 2(h)). In agreement, the expression of Slug, Twist1, and N-cadherin was decreased and the expression of E-cadherin was increased when Linc00261 was overexpressed in the HGSOC cells (Figure 2(i)). These results demonstrated that Linc00261 inhibited EMT phenotype of HGSOC.

### 3.4. Linc00261 Directly Bound to Inhibit miR-552 Expression

To explore the molecular mechanism of Linc00261 in HGSOC, StarBase V3.0 was used to predict the potential targets of Linc00261. The analysis revealed that a miRNA named miR-552 contained complementary sequence binding to Linc00261 (Figure 3(a)). To further verify whether Linc00261 directly binding miR-552, Linc00261-wt, or Linc00261-mut was cotransfected into HGSOC cell lines with miR-552 mimic, dual-luciferase reporter assay was carried out and found that the luciferase activity of Linc00261-wt group was significantly lower than Linc00261-mut group (Figure 3(b)). Then, the RNA pull-down experiment was used to validate the direct interaction between Linc00261 and miR-552. It displayed a remarkable increase of Linc00261 in miR-552-wt group than miR-552-mut group (Figure 3(c)). To explore the clinic correlation between Linc00261 and miR-552, qRT-PCR showed that Linc00261 expression was inversely correlated with the expression of miR-552 in HGSOC tissues (Figure 3(d)). Meanwhile, the result revealed that silencing Linc00261 expression significantly increased the expression level of miR-552 in CAOV3 cells (Figure 3(e)).

### 3.5. MiR-552 Promoted the HGSOC Progression via ATG10-EMT Pathway

Oncogenic miR-552 has been proved to play significant role in the progression of colorectal and hepatocellular carcinoma [37, 38]. However, the function of miR-552 on HGSOC is still unclear. So we ask whether miR-552 has similar tumor promoting function on HGSOC progression. Firstly, miR-552 expression was significantly upregulated in HGSOC tissue (Figure 4(a)). Moreover, qRT-PCR showed that miR-552 was notably overexpressed in ovarian cell lines (OVCAR3, OVCAR4, SNU119, CAOV4, and CAOV3) compared with normal ovarian epithelial cell line (FTSEC) (Figure 4(b)). Then, CCK-8 assay and transwell assay exhibited that miR-552 could promote HGSOC cell viability and migration (Figures 4(c) and 4(d)). To further explore the underlying mechanism of miR-552 on facilitating HGSOC progression, we performed bioinformatics analysis via targetscan database and discovered ATG10 was a potential target gene for miR-552 (Figure 4(e)). Then, dual-luciferase reporter assay was performed and results confirmed that miR-552 could interact with ATG10 (Figure 4(f)). Also, miR-552 could significantly inhibit expression level of ATG10 (Figure 4(g)). Furthermore, the correlation analysis of HGSOC clinical samples uncovered that the expression of ATG10 was negatively correlated with the expression of miR-552 (Figure 4(h)). These results suggested that miR-552 could combine and influence ATG10 expression. Given that ATG10 is an autophagy related gene and plays a tumor suppressive role through restraining the epithelial-mesenchymal transition (EMT) process [39]. Coincidentally, miR-552 played an oncogenic role by promoting EMT pathway in hepatocellular carcinoma [37]. Next, we want to know whether miR-552 regulates HGSOC progression via ATG10-EMT pathway. So the EMT related markers were detected and the results were showed that miR-552 inhibitor could reduce the mRNA and protein expression levels of Slug, Twist1, and N-cadherin (Figures 4(i) and 4(j)) and increase E-cadherin expression (Figures 4(i) and 4(j)). Meanwhile, silencing ATG10 could rescue the miR-552 inhibitor mediated EMT progression (Figures 4(i) and 4(j)). These data indicated that miR-552 promoted HGSOC progression via targeting ATG10 to induce EMT phenotype.

### 3.6. Linc00261 Suppressed the HGSOC Progression via miR-552-ATG10-EMT Pathway

Based on the above results, we speculated that Linc00261 could suppress EMT progression of HGSOC via targeting miR-552-ATG10 axis. Then, rescue experiments were determined to bear out the hypothesis. As shown in Figure 5(a), siLinc00261 or siNC was cotransfected with miR-NC or miR-552 inhibitor into HGSOC cells. We found miR-552 inhibitor could reverse the Linc00261 knockdown mediated expression level of miR-552 and ATG10. Furthermore, miR-552 inhibitor reduced the cell proliferation and migration capability after Linc00261 knockdown (Figures 5(b) and 5(c)). Also, the clinic correlation suggested that the expression of ATG10 was positively correlated with the expression of Linc00261 (Figure 5(d)). Furthermore, it is detected that miR-552 inhibitor could reverse the Linc00261 knockdown mediated EMT progression (Figure 5(e) and 5(f)). ATG10 knockdown could also rescue the Linc00261 overexpression restrained EMT progression (Figure 5(g) and 5(h)). Overall, these results demonstrated that Linc00261 suppressed EMT process by inhibiting miR-552-ATG10 axis, eventually preventing HGSOC tumorigenesis.

## 4. Discussion

A great number of studies exploring lncRNAs associated with diverse features in different tumor types demonstrated that lncRNAs play an essential role in all biological features of cancer cells [10, 40]. Recently, emerging research suggests that Linc00261 is a tumor suppressor in various cancers. For instance, Linc00261 inhibited non-small cell lung cancer cells progression via sponging miR-522 or suppressing EMT signaling [32, 41–43]. Also, Linc00261 has been recognized as a novel prognostic marker in many carcinomas, such as gastric cancer, pancreatic cancer, and hepatocellular carcinoma [44–48]. In this study, we report Linc00261, which is a tumor suppressor, inhibits HGSOC progression by competitively binding miR-552, elevating ATG10 expression, and then restrain EMT phenotype. We also find the expression of Linc00261 is decreased in HGSOC tissues and is further decreased in metastatic tumor tissues. Furthermore, it is showed that Linc00261 has pleiotropic effects on HGSOC cell proliferation and metastasis, and HGSOC tumorigenesis was suppressed by the Linc00261.

The lncRNA-miRNA-mRNA regulatory network was showed in many previous studies. At the posttranscriptional level, lncRNAs competitively sponge miRNAs, then resulting in suppression of targeted genes [49–52]. microRNAs (miRNAs/miRs) are 18–25 nucleotides in length, which are also a class of non-coding transcripts. microRNAs participate in diverse human diseases including many types of cancer [53]. A lot of studies have demonstrated that miR-552 acts as an oncogene in certain types of cancer [38, 54]. For instance, miRNA-552 promotes colorectal cancer progression via targeting DACH1 [55]. In osteosarcoma cell, miR-552 also facilitates tumor progression via targeting WIF1 [56]. Nevertheless, the relationship between miR-552 and lncRNA remains to be investigated. In our study, we find that Linc00261 interacts with miR-552 and inhibits miR-552 expression to increase ATG10 expression. As a result, the mRNA expression profile of EMT hallmarks, Slug, Twist1, N-cadherin, and E-cadherin, was influenced. It is widely recognized that EMT facilitates tumor invasion and dissemination [57]. Consistently, in our in vitro system, we all find that by restraining EMT phenotype, Linc00261 inhibits HGSOC tumorigenesis.

There are several limitations in this study. First, the number of collected HGSOC samples in our study is still limited. Second, the follow-up visit was not conducted to explore the association between the expression of LINC00261 and the prognosis of patients with HGSOC.

In conclusion, our results demonstrate that Linc00261 acts as a key negative regulator of HGSOC tumorigenesis. The findings of this study have significant implications regarding our understanding of HGSOC pathogenesis. The pleiotropic effects of Linc00261 on HGSOC progression suggest that Linc00261 might be an effective target for attractive therapies.

## Figures and Tables

**Figure 1:** Linc00261 was down-expressed in HGSOC. (a) Linc00261 expression was significantly lower in HGSOC tissues than in normal tissues. (b) LINC00261 expression in OVCAR3, OVCAR4, SNU119, CAOV4, CAOV3, and FTSEC cell lines. (c) Linc00261 expression was significantly downregulated in metastatic HGSOC tissue. Data are reported as means ± SD. ∗∗*P* < 0.01; ∗∗∗*P* < 0.001.

**Figure 2:** Linc00261 suppressed the proliferation and migration of HGSOC cells. (a) and (c) CCK-8 assays showed that Linc00261 inhibited HGSOC cells proliferation ability. (b) and (d) Transwell assays showed that Linc00261 inhibited HGSOC cells migration capacity. (e) Mice tumors were represented and linc00261 decreased tumor volumes. (f) and (g) The weights and volumes of the xenograft tumors derived from OVCAR3 cells stably expressing linc00261 or the negative control cells were examined. (h) and (i) The effect of linc00261 on EMT hallmarks mRNA expression by qRT-PCR. Data are reported as means ± SD. ∗*P* < 0.05; ∗∗*P* < 0.01.

**Figure 3:** Linc00261 directly bound to inhibit miR-552 expression. (a) A schematic outline of sequence sites of miR-552 targeted to LINCC00261 predicted by bioinformatic analysis. (b) Dual-luciferase reporter assay was carried out and found that the luciferase activity of Linc00261-wt group was significantly lower than Linc00261-mut group. (c) RNA pull-down assay was used to validate the direct interaction between miR-552 and LINC00261 in HGSOC cells. (d) The relationship between mRNA expressions of linc00261 and miR-552 in 23 pairs of HGSOC tissues. (e) The expression level of miR-552 was increased via silencing linc00261 expression. Data are reported as means ± SD. ∗∗*P* < 0.01; ∗∗∗*P* < 0.001.

**Figure 4:** MiR-552 promoted the HGSOC progression via ATG10-EMT pathway. (a) miR-552 expression was significantly higher in HGSOC tissues than in adjacent normal tissues. (b) The expression of miR-552 was detected in OVCAR3, OVCAR4, SNU119, CAOV4, CAOV3, and FTSEC cell lines by qRT-PCR. (c) CCK-8 assays showed that miR-552 promoted HGSOC cells proliferation ability. (d) Transwell assays showed that miR-552 elevated HGSOC cells migration capacity. (e) A schematic outline of sequence sites of miR-552 targeted to ATG10 predicted by bioinformatic analysis. (f) The expression of ATG10 was detected in miR-552 knockdown cells by qRT-PCR. (g) Dual-luciferase reporter assay was carried out to examine the luciferase activity of ATG10-wt group and ATG10-mut group. (h) The relationship between mRNA expressions of ATG10 and miR-552 in 23 pairs of HGSOC tissues was detected. (i) and (j) mRNA and protein levels of EMT markers were detected in miR-552 mimic, miR-552 inhibitor, siATG10 group, and miR-552 inhibitor plus siATG10 group by qRT-PCR. Data are reported as means ± SD. ∗*P* < 0.05; ∗∗*P* < 0.01; ∗∗∗*P* < 0.001.

**Figure 5:** Linc00261 suppressed the HGSOC progression via miR-552-ATG10-EMT pathway. (a) qRT-PCR validated that miR-552 inhibitor reversed the Linc00261 knockdown mediated expression level of miR-552 and ATG10. (b) and (c) miR-552 inhibitor reduced the cell proliferation and migration capability after Linc00261 knockdown via CCK-8 and transwell assays. (d) The relationship between mRNA expressions of ATG10 and Linc00261 in 23 pairs of HGSOC tissues was detected. (e) and (f) mRNA and protein levels of EMT markers were detected to verify the function of miR-552 inhibitor reversed the Linc00261 knockdown mediated EMT progression. (g) and (h) qRT-PCR and Western blot analysis were conducted to determine the function of ATG10 knockdown on Linc00261 overexpression mediated EMT progression. Data are reported as means ± SD. ∗*P* < 0.05; ∗∗*P* < 0.01; ∗∗∗*P* < 0.001.

## Data Availability

The datasets generated during and/or analyzed during the current study are available from the corresponding author on reasonable request.
